# Moderating role of compassion in the link between fear of Coronavirus disease and mental health among undergraduate students

This article has been retracted.

**DOI:** 10.3389/fpsyt.2022.990678

**Published:** 2022-09-06

**Authors:** Huichun Zhang, Saade Abdalkareem Jasim, Wanich Suksatan, Tawfeeq Abdulameer Hashim Alghazali, Rumi Iqbal Doewes, Abduladheem Turki Jalil, Indrajit Patra, Nermeen Singer, Virgilio E. Failoc-Rojas, Haydar Abdulameer Marhoon, Yasser Fakri Mustafa, Andrés Alexis Ramírez-Coronel, Abbas Abdollahi

**Affiliations:** ^1^Student Work Department of the Party Committee and Student Work Department, Inner Mongolia University of Technology, Hohhot, Inner Mongolia, China; ^2^Medical Laboratory Techniques Department, Al-Maarif University College, Al-Anbar-Ramadi, Iraq; ^3^Faculty of Nursing, HRH Princess Chulabhorn College of Medical Science, Chulabhorn Royal Academy, Bangkok, Thailand; ^4^Islamic University, Najaf, Iraq; ^5^Faculty of Sport, Universitas Sebelas Maret, Kentingan, Surakarta, Indonesia; ^6^Medical Laboratories Techniques Department, Al-Mustaqbal University College, Babylon, Hilla, Iraq; ^7^Independent Researcher, NIT Durgapur, West Bengal, India; ^8^Media and Children's Culture, Ain Shams University, Cairo, Egypt; ^9^Centro de Investigación en Medicina Traslacional, Universidad Privada Norbert Wiener, Lima, Peru; ^10^Information and Communication Technology Research Group, Scientific Research Center, Al-Ayen University, Thi-Qar, Iraq; ^11^Department of Pharmaceutical Chemistry, College of Pharmacy, University of Mosul, Mosul, Iraq; ^12^Laboratory of Psychometrics and Ethology and Health and Behavior Research Group, Universidad Católica de Cuenca, Ecuador; ^13^Universidad CES, Medellín, Colombia; ^14^Universidad Nacional del Ecuador Cuenca, Ecuador; ^15^Universidad de Palermo, Argentina; ^16^Department of Counseling, Faculty of Education and Psychology, Alzahra University, Tehran, Iran

**Keywords:** fear of COVID-19, mental health, self-compassion, partial least squares, university students

## Abstract

**Background:**

The societal challenges presented by fear related to the coronavirus disease (COVID-19) pandemic may present unique challenges for an individual's mental health. However, the moderating role of compassion in the relationship between fear of COVID-19 and mental health has not been well-studied. The present study aimed to explore the association between fear of COVID-19 and mental health, as well as test the buffering role of compassion in this relationship.

**Methods:**

The participants in this study were 325 Iranian undergraduate students (228 females), aged 18–25 years, who completed questionnaires posted on social networks via a web-based platform.

**Results:**

The results showed that fear of COVID-19 was positively related with physical symptoms, social function, depressive symptoms, and anxiety symptoms. The results also showed that compassion was negatively associated with physical symptoms, social function, depressive symptoms, and anxiety symptoms. The interaction-moderation analysis revealed that compassion moderated the relationship between fear of COVID-19 and subscale of mental health.

**Conclusion:**

Results highlight the important role of compassion in diminishing the effect of fear of COVID-19 on the mental health (physical symptoms, social function, depressive symptoms, and anxiety symptoms) of undergraduate students.

## Background

Coronavirus disease (COVID-19) spread rapidly across countries, causing great financial and human losses as well as concern and fear among the general public (1). At the time of writing, more than 90 million people worldwide have been infected with the disease since the initial outbreak in Wuhan, China on December 2, 2019, and more than 1.9 million have died from the virus (2). Iran has one of the highest number of infected cases per population (3). The first case of COVID-19 in Iran was identified in March 2020; to date, more than seven million people have been infected and more than 140,000 people have died from the virus in Iran.

As the scope of the issue became clearer during the onset of the pandemic and a state of emergency was declared by the WHO, governments gradually started introducing policies such as quarantine and social distancing (4). Despite the positive physical health aspects of enforcing such policies, there have already been negative psychological consequences, including increased levels of anxiety and stress (5). These consequences may have severe and long-term effects on the mental health of various groups of people, particularly young people, as they are one of the segments of society most vulnerable to the psychological effects of the pandemic (6). Due to the closure of universities and businesses, mandatory stay at home orders, reduced communication and social support, as well as family financial issues, young people are more vulnerable to unpleasant feelings, including fear and uncertainty about the future (7). A study of young people in Iran showed that their fear and anxiety about the spread of the virus have increased slightly since the first wave (September 2020) (8). The results of previous studies have shown that the implementation of quarantine exacerbated the symptoms of depression, anxiety, loneliness, and sleep problems in the general population (9, 10). While most recent research on the psychological effects of the virus and quarantine has been focused on general population, medical staff, in particular nurses (11–14), it is critical that the mental health of undergraduate students not be forgotten. Previous studies have conducted on undergraduate students' well-being, anxiety, and depression during the COVID-19 pandemic (15–19). However, the moderating role of compassion in the relationship between fear of COVID-19 and mental health among undergraduate students has not been studied. Therefore, the aim of this study is to understand the buffering role of compassion in the relationship between fear of COVID-19 and mental health among undergraduate students.

Numerous studies have shown that life events may influence the well-being and mental health of people (20–22). The concept of well-being and mental health is not just the absence of individual mental illness, but rather the ability for an individual to thrive and be mentally well-adjusted in order to face obstacles. Well-being allows people to experience a rewarding, productive, meaningful, and virtuous life (2). The General Health Questionnaire (GHQ-28) is a commonly used instrument for assessing mental health and psychosocial well-being (23). In this study, the GHQ-28 was used to measure mental health (24). The GHQ-28 covers four main areas) somatic symptoms, social dysfunction, anxiety symptoms, and depression symptoms). In this study, four areas are examined separately instead of the overall score for mental health. The GHQ-28 examines disruptions in normal function that result in an incapacity to engage in usual healthy activities.

The basis of this study is whether compassion can play a moderating role in the relationship between fear of COVID-19 and mental health among undergraduates. A moderator can strengthen or weaken a relationship and act as a buffer. In this study, we examined the joint relation of fear of COVID-19 and a potential moderator (compassion), to mental health in undergraduate students. Compassion has attracted the attention of researchers as one of the newest structures of the positive psychological approach. An agreed upon definition in the literature suggests compassion is the attention given to the strengths of individuals effective in improving their mental health (25–27). Studies have shown that compassion plays a supportive role against perceived stress and helps individuals to experience less perceived stress during the ongoing COVID-19 pandemic (28–30). Recent studies also are supportive of the benefits of compassion for emotional regulation (31), increasing resilience (32), efficient intra- and inter-personal interactions (33), and mental health (29). Being compassionate to others and the ability to be open to receiving compassion from others mitigate the symptoms of depression and anxiety (34). Recent studies have shown that depression, stress, and anxiety make people vulnerable to infection after being exposed to the coronavirus and decrease the immune system's response to immunizations (35, 36). Therefore, study about protective factors that might increase the mental health effects of the COVID-19 pandemic is imperative and it is one of the priorities of mental health science. Compassion is vital in regulating one's own and others' emotions, more effective social relationships, and maintaining mental health of individuals, and it may be a protective factor against the impact of fear of COVID-19 on mental health. Although previous studies have addressed the supportive role of compassion. Little attention has been paid to the moderating role of compassion between fear of COVID-19 and mental health in undergraduate students and this study aims to address this gap in the literature.

This study employed a new compassion scale derived from the study of Neff on self-compassion scale (37). Neff (38) pointed to three aspects of self-compassion: self-kindness, common humanity, and mindfulness. Self-kindness entails being decent and kind to oneself, rather than causing inner pain and being self-critical. Common humanity is being aware of the common tragedy and suffering of human beings. Having this aspect of self-compassion allows the individual to understand how human beings are equal in experiencing the concept of suffering, for instance during a global pandemic. Finally, mindfulness entails living in the present moment with a clear and unambiguous acceptance and understanding of emotions (38). The definition of the compassion scale is similar to the self-compassion scale, except that the compassion scale focuses more on being compassionate to others and less uncompassionate toward others in terms of emotional response, cognitive perception, and attention to the suffering of others. The compassion scale focuses more on the general suffering of others' lives, kindness to others, caring toward others, and supporting others. Common humanity in compassion scale is defined as an individual with high levels of sense of connection with people who experience hardship and suffering. Mindfulness in compassion scale involves an interpersonal understanding of the suffering of others and paying attention and empathizing with the suffering of others (37).

When people are under stress specifically in the situation of COVID-19 pandemic, caring and supporting themselves and others have strong psychological and physiological effects. Therefore, compassion can be considered as an intra- and inter-personal process that can help both individuals and others to have less fear of COVID-19 and experience higher levels of mental health in a social interactional context (29). Research shows that compassion as a potential coping method, reduces fear and stress, regulates emotions, and promotes mental health and well-being (39, 40). While greater compassion is associated with lower levels of fear and stress, no study to date has specifically examined the relationship between compassion, fear of the COVID-19 pandemic, and mental health outcomes among Iranian undergraduate students.

The purpose of this study was two-fold. First, the present study examined the relationship between fear of COVID-19, mental health, and compassion in a sample of undergraduate students. Second, the study examined whether compassion moderated the relationship between fear of COVID-19 and mental health. This study therefore hypothesized (a) a negative relationship between fear of COVID-19 and mental health and (b) predicted that compassion would be a moderator between fear of COVID-19 and mental health among undergraduate students.

## Methods

### Participants

The statistical population of the study consisted entirely of undergraduate students at Tehran University and Islamic Azad University Science and Research Bran, Tehran in the first half of the 2020–2021 academic year (20 December 2020 to February 2021). The number of potential participants in this study was around 1,500 undergraduates. According to Kline (41), sample sizes between 200 and 500 are needed when using structural equation modeling (SEM). Data from 335 participants were collected by using an available sampling method. After 10 questionnaires were removed due to response deficiencies, surveys from 325 participants (228 females and 97 males) remained for data analysis. Of the total participants, 259 (80%) were single and 66 (20%) were married. The ages of the participants ranged from 18 to 25 years old, with a mean age of 21.85 (*SD* = 5.42). Participants were from public universities (298 students) and private universities (27 students). Roughly half of the students were studying in the medical field (*N* = 146; 45%), 94 (29%) studied in technical fields, and 84 (26%) were students in various social science fields. One hundred (30%) students were in their first year of university, 120 (37%) students were in their second year of university, 60 (18%) were in their third year of university, and 45 (15%) were in their final year of university.

### Procedure

The current study's process and research materials were approved by Alzahra University's ethical committee (Reference Number: 1401/05/15). Google Forms was used to design and present questionnaires and the link to the survey was provided to potential respondents via various social networks (i.e., WhatsApp and Telegram). The required permit was obtained from Alzahra University and Islamic Azad University Science and Research Bran to comply with ethical standards and the subjects were assured that their data and information would remain confidential. The researchers of this study invited undergraduates via WhatsApp and telegram social networks to complete the link questionnaires. Participants signed electronically informed consent and could request the option to obtain the results of the research after the study had concluded. To be eligible to participate, participants had to be between the ages of 18 and 25, be pursuing a bachelor's degree, and be ready to participate in the study. Participants were excluded if they did not agree to participate.

### Measures

#### The general health questionnaire

The General Health Questionnaire (GHQ) is a 28-item questionnaire used to measure a person's mental state (24), and includes the subscales of physical symptoms (sample item: *Been getting any pains in your head?*), anxiety symptoms (sample item: *Been feeling nervous and strung-out all the time?*), social functioning (sample item: *Been able to enjoy your normal day-to-day activities?*), and depressive symptoms (sample item: *Been feeling that life is not worth living?*). Each subscale has seven items, which are measured on 4-point Likert scale (0 = never, 3 = always). In this study, higher scores indicate poorer mental health. Taghavi (42) found the survey had very good internal validity (Cronbach's alpha = 0.91) and sufficient reliability with a sample from Iran.

#### The fear of COVID-19 scale

This scale consists of seven items and assesses the extent and severity of fear of COVID-19 (43). Participants respond to the survey on a 5-point Likert scale (1 = strongly disagree, 5 = strongly agree), with higher scores suggesting a greater fear of COVID-19. A sample item is “*I am most afraid of coronavirus.”* The scale was found to have good reliability (Cronbach's alpha = 0.82) (43).

#### The compassion scale

The Compassion Scale (CS) is a 16-item scale that measures an individual's compassion (37). This questionnaire consists of four subscales: Indifference (sample item: *I am unconcerned with other people's problems*); Kindness (*sample item: I like to be there for others in times of difficulty*); Mindfulness (sample item: *I listen patiently when people tell me their problems*); and Common humanity (sample item: *I realize everyone feels down sometimes, it is part of being human*). Each subscale containing four items. Participants answer the questionnaire on a 5-point Likert scale (1 = almost never, 5 = almost always), with higher scores specifying higher levels of compassion. The Brislin method was used to translate the measure into Persian (44). Results from this study showed appropriate content validity (CVI = 0.86) and face validity (Impact score = 1.7); the measure also had very good reliability (Cronbach's alpha = 0.91).

### Statistical method

Structural Equation Modeling analysis with Partial Least Squares in the PLS3 software (version 3.2.3) was used in response to the research objectives (45). The advantage of using the SEM analysis method over other common methods such as regression analysis and factor analysis is that SEM can be used to analyze multiple relationships and factor analyses simultaneously. The partial least squares method also provides the highest estimate of the coefficient of determination for the endogenous variable predicted by the exogenous variables (46). Effect size [*f*^2^; when the values of *f*^2^ are 0.02, 0.15, and 0.35, Cohen classifies *f*^2^ as small, medium, and large effect size, respectively (47)] and Stone–Geisser [*Q*^2^; when the values of *Q*^2^ are 0.02, 0.15, and 0.35, Henseler and colleagues classify *Q*^2^ as small, medium, and large, respectively (48)] were all evaluated for the structural model (46). A higher value of *f*^2^ indicates greater effect size of the exogenous variable on the endogenous variable and a higher value of *Q*^2^ indicates large predictive relevance of exogenous variable.

## Results

### Measurement model

For the measurement model, the Average Variance Extracted (AVE) was employed to assess the convergent validity, the Composite Reliability (CR) was employed to assess construct reliability, and the Variance Inflation Factor (VIF) was employed to assess discriminant validity (46). Acceptable cut-off scores for AVE, CR, and VIF are 0.5, 0.7, and <5, respectively (46). As seen in Table 1, the research variables have satisfactory convergent validity, construct reliability, and discriminant validity. As seen in Table 1, the participants' total scores in GHQ-28 were <23 (the cut-off for total score of GHQ-28 is 24), indicating good health (23). The mean score for the CS in this study was (56.12) greater than the mean score for the CS in the main study (37, 54). As seen in Table 1, the means and standard deviations for indifference, kindness, mindfulness, and common humanity were 14 ± 3.21, 15 ± 2.21, 12 ± 2.87, and 10 ± 2.54, respectively. The mean score for the fear of COVID-19 scale in this study was (26.35) same as the mean score for the fear of COVID-19 scale in the main study (43).

**Table 1:** Values of composite reliability, average variance extracted, variance inflation factor, mean, and standard deviation.

**Variable**	**Cronbach's alpha**	**CR^a^**	**AVE^b^**	**VIF^c^**	***M***	***SD***
General Health Questionnaire	0.93	0.94	0.57	–	18.34	3.66
Physical symptoms	0.92	0.91	0.58	–	13	2.12
Social function	0.91	0.92	0.55	–	12	2.18
Depressive symptoms	0.9	0.89	0.56	–	13	3.15
Anxiety symptoms	0.92	0.93	0.58	–	14	3.41
Compassion	0.91	0.89	0.51	1.04	56.12	3.54
Indifference	0.89	0.87	0.52	–	14	3.21
Kindness	0.9	0.89	0.53	–	15	2.21
Mindfulness	0.89	0.86	0.56	–	12	2.87
Common humanity	0.89	0.87	0.54	–	10	2.54
Fear of COVID-19	0.87	0.88	0.59	1.04	26.35	5.55

a Composite reliability.

b Average variance extracted.

c Variance inflation factor.

### Structural model

The results of the path analysis showed that compassion negatively associations with physical symptoms (β = −0.365, *t* = 2.85, *p* < 0.001), social function (β = −0.389, *t* = 3.11, *p* < 0.001), depressive symptoms (β = −0.462, *t* = 3.45, *p* < 0.001), and anxiety symptoms (β = −0.475, *t* = 3.24, *p* < 0.001). The result of path analysis also showed that fear of COVID-19 positively associations with physical symptoms (β = 0.353, *t* = 2.74, *p* < 0.001), social function (β = 0.469, *t* = 3.88, *p* < 0.001), depressive symptoms (β = 0.469, *t* = 3.55, *p* < 0.001), and anxiety symptoms (β = 0.480, *t* = 3.26, *p* < 0.001; see Figure 1).

**Figure 1:** Structural model for general health questionnaire.

*R*^2^ shows the amount of variance in the endogenous variable (physical symptoms, social function, depressive symptoms, and anxiety symptoms) via the exogenous variables (compassion and fear of COVID-19). The result showed that by increasing one unit in the exogenous variables (compassion and fear of COVID-19), 13.3%, 21.7%, 20%, and 30.3% variation occurred in the endogenous variables (physical symptoms, social function, depressive symptoms, and anxiety symptoms). The effect size (*f*^2^) was used to assess the influence of the exogenous variables (compassion and fear of COVID-19) on the endogenous variable (physical symptoms, social function, depressive symptoms, and anxiety symptoms). In this study, the effect size of compassion and fear of COVID-19 were 0.55 and 0.35, respectively, which indicate the magnitude of the large effect size of both exogenous variables on endogenous variables (physical symptoms, social function, depressive symptoms, and anxiety symptoms). *Q*^2^ was used to assess the predictive value of the endogenous variables (physical symptoms, social function, depressive symptoms, and anxiety symptoms). In the present study, the values of *Q*^2^ for physical symptoms, social function, depressive symptoms, and anxiety symptoms was 0.58, 0.61, 0.68, and 0.71, indicating large predictive relevance of subscale of mental health (*Q*^2^ >0.35).

### Moderation test of compassion

The interaction-moderation approach was used to investigate the moderating role of compassion in the association between fear of COVID-19 and mental health (physical symptoms, social function, depressive symptoms, and anxiety symptoms). The result of the interaction effect of compassion and fear of COVID-19 showed a significant negative association with physical symptoms (β = −0.101, *t* = 1.99, *p* = 0.03), social function (β = −0.134, *t* = 2.18, *p* < 0.05), depressive symptoms (β = −0.128, *t* = 2.08, *p* < 0.05), and anxiety symptoms (β = −0.131, *t* = 2.16, *p* < 0.05). Thus, compassion played a moderating role on the relationship between fear of COVID-19 and physical symptoms, social function, depressive symptoms, and anxiety symptoms. The moderation effect sizes for physical symptoms, social function, depressive symptoms, and anxiety symptom were 0.41, 0.49, 0.47, and 0.51, respectively. Henseler (49) classified moderation effect size as weak, moderate, and strong when the values are 0.02, 0.15, and 0.35, respectively.

## Discussion

The present research was carried out to gain a deeper insight into the psychological problems caused by the ongoing COVID-19 pandemic and to explore the relationship between fear of the virus, mental health, and compassion in an Iranian sample of undergraduate students during the university closure due to quarantine.

This study investigated the moderating role of compassion in the relationship between fear of the COVID-19 and mental health. Similar to previous research (50, 51), the present study demonstrated that greater fear are associated with greater levels of somatic symptoms, social dysfunction, anxiety symptoms, and depression symptoms in undergraduate students. The findings of the current study showed that higher levels of fear of COVID-19 were associated with higher levels of somatic symptoms, anxiety symptoms, lower social functioning, and depressive symptoms (as subscales of the GHQ). Thus, fear of COVID-19 is associated with increased somatic symptoms, social dysfunction, anxiety symptoms, and depression symptom. Our findings are in line with previous studies showing that fear of COVID-19 is associated with poorer mental health (29, 30). Given the ongoing state of the pandemic, the findings demonstrate the importance of identifying a construct (compassion) that moderates the negative impact of fear of COVID-19 on somatic symptoms, social dysfunction, anxiety symptoms, and depression symptoms of undergraduate students who experience higher levels of fear of COVID-19. The results of the SEM analysis showed that compassion is a construct that reduces the negative impact of fear of COVID-19 on mental health issues. Our findings suggest that greater levels of compassion associated with lower levels of fear of COVID-19 and greater levels of mental health in Iranian undergraduate students. As undergraduate students are subjected to more psychological stressors during the COVID-19 pandemic (e.g., social isolation, fear of quarantine) (52), the results of this study hold promise for alleviating some negative psychological impacts. The caveat is that this study was not causal, and the direction of influence cannot be determined, i.e., more naturally compassionate individuals likely have better mental health and less fear of the pandemic.

The results of the present study demonstrated that compassion has a significant moderation role between fear of COVID-19 and mental health among undergraduates. Various studies have provided evidence for the effectiveness of compassion in reducing psychological symptoms such as fear, stress, depression, and suicide, and increasing positive emotions (53, 54). One study has found that such individuals are kinder to themselves, and are less likely to be self-critical and ruminate on negative events (55).

Consistent with prior research, the results of the present study demonstrated that compassion also has a significant relationship with mental health (56). The findings showed that compassion was negatively associated with the four measured components of mental health (physical symptoms, anxiety symptoms, social functioning, and depressive symptoms). According to study findings, the component of indifference by itself can improve undergraduate students' mental health. The sample item of the indifference component is “I don't concern myself with other people's problems; this item is reverse coded.” People who score high in the indifference component are likely to have compassionate responses to the pain and suffering of others. As we know, one of the components of mental health is having a sense of empathy with others, and people who have more empathy are more likely to have better quality interpersonal relationships and they are more likely to experience greater levels of mental health (57). Results of the study found that the component of kindness by itself is effective in increasing the mental health of undergraduate students. In other words, people with high levels of kindness experiences may have better mental health by having a kind and non-judgmental attitude toward themselves. Common humanity may help individuals to reduce their COVID-19 fears. In other words, COVID-19 fears are experienced as a common, shared experience, which may reduce isolation and discomfort and increase one's well-being. Note that the mindfulness aspect of compassion was found to decrease mental occupation, and allow individuals to accept experiences and emotions without avoiding and over-identification. Mindfulness also helps individuals neither avoid nor get lost in suffering of self and others and to have more acceptance of the suffering of self and others. Mindfulness helps individuals to live in the present and do not be involved in the past events or future thoughts (37). As a result, by reducing an excessive focus on fear of COVID-19, negative emotions may decrease, while positive emotions and a focus on the present (e.g., the here and now) may increase. Compassion includes compassion for others and from others, which can help individuals to have effective social relationships, mitigate the symptoms of anxiety and depression, and may regulate emotional processes that may contribute to better mental health during the COVID-19 pandemic (29). Based on previous studies (29, 30) and the results of the current study, it is confirmed that compassion plays an important role as a significant protective factor and moderating factor between fear of COVID-19 and mental health difficulties.

## Implications of study

This study provides support for the moderating role of compassion in the relationship between fear of COVID-19 and mental health among undergraduates. Therefore, the accurate assessment of fear of COVID-19, compassion, and mental health in undergraduate students is essential for educational psychologists and clinicians. It has been thoroughly demonstrated that compassion plays a key role in reducing fear of COVID-19 and improving mental health. Therefore, it is plausible that interventions that increase compassion may increase the mental health of undergraduate students.

## Limitations of study

There were several limitations to the present study. First, this study is a cross-sectional study, which limits the scope and long-term validity of the results. It is necessary to conduct longitudinal studies in the field of psychology during the ongoing pandemic to obtain more valid data. The second limitation was related to the study sample. As the study population consisted solely of undergraduate students from a single country, caution should be exercised in generalizing the results to other populations. It is suggested that other studies be performed to investigate the negative psychological effects of the pandemic on other age groups. It is also important to examine other structures that may mediate the relationship between COVID-19 fear and mental health. In this regard, comparing gender differences could be a valuable aid in identifying the impact of COVID-19 on the mental health dimensions of different sexes. Because increasing levels of mental health and life satisfaction influence the academic and occupational performance of undergraduate students, it will be valuable for future studies to determine whether a good quality of life impacts other mechanisms such as academic and occupational satisfaction and motivation during the COVID-19 outbreak.

The findings of this study indicate that higher levels of compassion moderate the relationship between fear of COVID-19 on mental health among Iranian undergraduate students.

## Data availability statement

The datasets presented in this study can be found in online repositories. The names of the repository/repositories and accession number(s) can be found below: https://doi.org/10.6084/m9.figshare.13654133.v1.

## Ethics statement

The Ethics Committee of the Alzahra University (IR/11/12/1399) approved the study procedure and informed consent was obtained from the participants. All methods have been carried out in accordance with relevant guidelines and regulations.

## Author contributions

HZ, AA, SJ, WS, TH, RD, and AJ designed the study, collected the data, and writing the draft of manuscript. IP, NS, VF-R, and HM helped to write the manuscript, provided the comments to improve the quality of manuscript, and responded to the reviewers' comments. YM and AR-C analyzed the data, reviewed the manuscript, and answered to the reviewers' comments. All authors contributed to the article and approved the submitted version.

## Conflict of interest

The authors declare that the research was conducted in the absence of any commercial or financial relationships that could be construed as a potential conflict of interest.

## Publisher's note

All claims expressed in this article are solely those of the authors and do not necessarily represent those of their affiliated organizations, or those of the publisher, the editors and the reviewers. Any product that may be evaluated in this article, or claim that may be made by its manufacturer, is not guaranteed or endorsed by the publisher.
